The article "A Deep Learning-Based TE Method for MSs' Mental Health Analysis" was retracted in 2023. Reasons: signs of a paper mill; suspected computer-generated content; unreliable results or conclusions; concerns about the data.

# A Deep Learning-Based TE Method for MSs' Mental Health Analysis

**DOI:** 10.1155/2022/1420542

**Published:** 2022-09-29

**Authors:** Ranxin Tao

**Affiliations:** School of Marxism, Zhengzhou College of Finance and Economics, Zhengzhou Henan 450000, China

## Abstract

Teaching evaluation (TE) is of great significance in education and can judge the value and appropriateness of the curriculum, which is a distinguished part of the educational work. Compared with other courses focusing on imparting knowledge, mental health not only imparts psychological knowledge but also cultivates Marxism students' (MSs) ability to adjust psychology and maintain mental health. Therefore, the evaluation of this course has a special character. As the unity of scientific world outlook and values, Marxism can promote students' mental health. When assessing students' ability to maintain mental health, the influence of Marxism should be taken into account. In this study, we first established an evaluation index system in line with the actual mental health considering the influence of Marxism and put forward a deep memory network with prior information (PI-DMN) to realize the aspect-based sentiment analysis (ABSA) of the student evaluation text. Combined with students' scoring of the course, the sentiment analysis results are used as the input dataset of LSTM model to realize the TE of mental health course. The data analysis exposes that Marxism can promote mental health, and the empirical analysis reveals that the accuracy of TE can be improved by considering the sentiment analysis of comment texts and can also be improved to a certain extent after aspect labeling of the dataset.

## 1. Introduction

Objective and scientific evaluation of courses is the premise of improving teaching quality. Students are the direct audience of teaching services, so students' feedback on teaching has important reference significance for understanding and improving teaching. TE is an extensively applied method to collect students' feedback on the quality of curriculum teaching [1, 2]. It is the evaluation made by students on the teaching attitude, teaching method, teaching content, teaching effect, and other aspects of the course or teachers according to certain evaluation indicators [3, 4]. TE can better reflect the detailed information of students' satisfaction with all aspects of teaching, which can be used as an important method for teaching management to measure the teaching effect and can also be used to help teachers to improve teaching [5, 6]. Although the existing teaching effect evaluation methods have an active effect on promoting the improvement of teaching level and quality, there are certain shortcomings: the evaluation results are influenced by human factors; some of them are only unilaterally evaluated by students' performance, which is obviously one-sided; due to the dynamic interaction of teaching, the diversity of influencing factors, and the variability of influencing factors, it is actually a nonlinear mapping problem with relatively complex structure; and the evaluation results cannot be expressed by simple mathematical analysis formula [7]. Therefore, it is easy to lead to distortion and bias in evaluation results, and unreasonableness still exists. Mental health is not an ordinary subject course, which is not only to teach psychological knowledge but also to cultivate students' ability to maintain mental health. Therefore, the evaluation of this course is special.

Sentiment analysis techniques have been applied by many researchers in the field of education, especially for student feedback, because of their good ability to handle unstructured data such as text [8]. Text sentiment analysis is the process of collecting, processing, analyzing, generalizing, and reasoning about subjective texts with emotional overtones [9] and involves various research fields such as artificial intelligence, machine learning, data mining, and natural language processing [10, 11]. Sentiment analysis is a typical problem in text classification in the field of natural language processing, that is, classifying the text to be analyzed into one of its categories [12, 13]. Text sentiment analysis is generally applied to study people's emotions, opinions, or attitudes towards goods, services, events, and other research objects, and it can realize the automatic processing of text data, so it is widely used in e-commerce comments, public opinion analysis, online education, and other fields. In the current research, curriculum scoring is applied more, but there is less text analysis of students' curriculum comments, and curriculum comments contain students' true attitudes. Therefore, this paper integrates emotional analysis of curriculum comments into a part of teaching evaluation.

In recent years, DL has achieved good performance in the fields of data mining, natural language processing, and machine translation [11]. The core idea of DL is “a neural network that simulates the human brain for learning and analysis.” Its concept comes from the study of artificial neural networks [14, 15]. If we teach computers to recognize many cards like children, then we need to let computers first look at these cards repeatedly. After cyclic learning and training, when the same cards are given, the computer can recognize them directly [16, 17]. The same is true for emotional analysis based on DL; by training a large number of datasets, let the machine summarize the rules in the brain. When it sees a sentence that conforms to this rule next time, it can directly judge the emotional score of the sentence [18]. In the DL model, word embedding method is used to refrain from the processing difficulties generated by uneven text length, and the DL model can also accurately capture abstract features to avoid cumbersome feature extraction [19, 20]. These advantages make DL play a significant role in text processing and have become the mainstream method of emotion analysis [21, 22]. Therefore, utilizing emotion analysis technology based on DL to mine students' emotional tendencies from a large number of data is the key to fully realize TE. This study first establishes an evaluation index system that conforms to the reality of mental health and proposes a PI-DMN model to realize the aspect-based emotion analysis of students' evaluation text. Combined with students' scoring of the course, it is used as the input dataset of LSTM model to realize the teaching evaluation of mental health courses.

## 2. Related Work

Due to the important research significance of TE, increasing scholars begin to pay attention to this field and put forward some effective methods. Wadawadagi and Pagi [23] proposed a stacking integration method, which combines the output of deep learning with the feature-based machine learning model to predict the intensity of emotion and emotion. Bahdanau et al. [24] proposed a method of automatically building a domain specific emotional dictionary to avoid emotional ambiguity. However, the efficiency of feature engineering of these manually set rules is very low, which seriously affects the accuracy of emotion classification. Akhtar et al. [25] used various machine learning methods to automatically extract emotional information from student teaching evaluation, compared their performance, and then applied them to the student teaching evaluation of university teaching management system. Yanyan et al. [26] used a variety of text representation methods, combined with a variety of supervised learning algorithms, reinforcement learning methods, and DL models for comparative analysis. Chiu-Wang et al. [27] designed a decision support system, using a variety of methods such as deep neural network, RNN with attention mechanism, and LSTM to analyze the Chinese text opinions of the teaching evaluation questionnaire. Cabada et al. [28] introduced the DL architecture that can be used for educational emotion analysis. The convolutional neural network model with long-term and short-term memory has achieved a high classification accuracy. Zheng et al. [29] proposed an end-to-end antagonism memory network, which extracts common features of source and target domains by adding AMN model and using adversarial training automatically. Gomez et al. [30] build a comprehensive online teaching evaluation tool based on the online learning environment, linking the role of teachers, teacher performance, demographic characteristics of students, and teaching effects. Barteit et al. [31] study the quality of online education in the medical field in low-income countries and believe that most countries still need to take measures to explore more effective and reliable online course evaluation methods. Calderon and Sood [32] evaluate the quality of online courses through three dimensions: teaching situation, interactive communication quality, and metalearning. In the above research, the teaching evaluation do not comprehensively consider the emotion of the course review text and the course score, and no corresponding indicators are put forward specifically for the course of mental health. This paper proposes a new teaching evaluation method to solve the above problems.

## 3. Teaching Evaluation Method Based on DL

### 3.1. Assessment Index of Mental Health Course for Students Majoring in Marxism

The establishment of comprehensive assessment index system of instructional curriculum is the basis of comprehensive assessment [33, 34]. Starting from many interfering factors of teaching effect, this study constructs a comprehensive evaluation index system on the basis of analyzing and summarizing many relevant documents of teaching assessment. The rational formulation of the comprehensive evaluation index system of teaching effect is of great significance for accurately measuring the value of course teaching effectiveness and also provides an important reference for teaching reform decision-making.

Mental health education course is a comprehensive course integrating psychological knowledge, strengthening psychological experience, and training psychological adjustment ability. It is not an ordinary discipline curriculum, but more than the transmission of psychological knowledge, it is more important to promote the overall development of students' psychological quality. On the basis of the study of mental health knowledge and the cultivation of mental health awareness, by giving full play to students' subjectivity, students can obtain direct inner experience through their own practical activities and cultivate various abilities such as self-cognition and self-adjustment. Therefore, the evaluation index of mental health course should be different from other courses, and the evaluation index should consider the improvement of the course on the students' psychological state. Marxism as a philosophy, students of this major should learn to see and solve problems through a Marxist perspective. Marxism is the unity of scientific outlook on life and values, which can guide students to establish a positive attitude towards life. Marxism advocates looking at problems from the perspective of development, which can cultivate a positive thinking mode and promote mental health to a certain extent. Therefore, the influence of Marxism on students' mental health should be considered; whether students can reasonably use the principles of Marxism to solve the troubles in life should also be included in the evaluation index of students' ability to maintain mental health.

On the basis of the comprehensive analysis of the interfering factors of course teaching effect evaluation, combined with the characteristics of teaching reform, through investigation of a large number of data and text materials and consultation of experts, this study established a comprehensive assessment index system for the teaching effect of mental health course. The index system mainly includes five first-level indicators, teaching attitude, teaching effect, teaching method, lecture effect, psychological improvement, and the second-level indicators that make up them, as shown in Table 1. Course indicators are obtained through an electronic questionnaire. Each secondary evaluation indicator in the questionnaire is set to 5 levels of “strongly agree, agree, general, disagree, and strongly disagree,” and the corresponding scores are “5, 4, 3, 2, and 1,” respectively.

### 3.2. Aspect-Based Sentiment Analysis of Teaching Review Text Based on PI-DMN

Compared with scoring method, teaching review text can better reflect the true attitude of students. Aspect-based sentiment analysis (ABSA) is a fine-grained sentiment classification task that aims to determine the sentiment polarity of a particular aspect, which consists of two subtasks: the aspect word extraction and the aspect-level emotion classification. For example, through the course comment “Teacher Li's class inspires me, but he rarely communicates with students,” it can be seen that the comment expresses positive emotions in terms of “enlightenment” while negative emotion in the aspect of “Teacher-student interaction.” This study proposes an emotion recognition method based on PI-DMN. Combined with the prior knowledge of comments, we achieve the ABSA of teaching review text in five aspects: “teaching attitude,” “teaching effectiveness,” “teaching method,” “lecture effect,” and “psychological improvement.”

#### 3.2.1. Deep Memory Network

The traditional RNN model has weak memory ability of hidden state and attention mechanism and cannot store a large amount of semantic information, so it is easy to lose important semantic information in the primitive sentence. The memory network (MN), on the other hand, is designed to store contextual information about a sequence in a separate memory module, to be read and used when necessary, and is first utilized in question-and-answer systems. MN is a machine learning framework that is essentially an inference process with a long-term memory structure, which consists of four parts, including an input module, a generalization module, an output module, and a response module, as shown in Figure 1.

Deep memory network (DMN) is an extension of the base model of MN, which contains more hidden units than the shallow MN, thus capturing more abstract features. And the model learns a better fit function and exhibits better memory capabilities. The DMN uses an external memory module to model the semantics of the original text and then superimposes the input and output layers of the model to extract as much abstraction relationship as possible between the text and the input problem. The structure of the four-layer end-to-end DMN model is shown in Figure 2.

Based on DMN, this study proposes a deep memory network model incorporating prior knowledge and applies it to aspect-level sentiment analysis of student teaching evaluation. Using prior knowledge instead of the question as the input to the network, the answer to the question is judged from the information in the memory constructed by the context of the comment. The LSTM unit is applied to update the prior knowledge, which can correct the prior knowledge and complete ABSA when aspect labels are not available for the comments. As shown in Figure 3, the PI-DMN model consists of the following four processes: text preprocessing and word embedding, contextual semantic modeling, sentiment representation, and sentiment recognition.

#### 3.2.2. Text Preprocessing and Word Embedding

The quality of text processing directly affects the accuracy of machine learning. The text data is cleaned by regular expressions firstly. After removing the invalid information, the text needs to be segmented using word segmentation techniques to improve the efficiency of sentiment analysis. In this study, we utilize the Jieba library in Python to implement the text segmentation. Finally, we remove the deactivated words in the text that do not have actual meaning but only serve to connect the text, so as to improve the accuracy of sentiment analysis and reduce the amount of computation.

Word embedding is a method to transform words in a text into numeric vectors. Teaching evaluation text is unstructured data that cannot be recognized by computers. In order to use standard machine learning algorithm to analyze them, these words need to be converted into numeric vectors and utilized in digital form as input. The essence of word embedding is to learn a mapping that converts words into unique corresponding vectors, mainly including one hot coding, continuous bag-of-words (CBOW), and skip-gram model. One-hot encoding uses *n*-dimensional vectors to encode *n* words, each word has only 1 element in its corresponding vector position, and the rest elements are 0. When the vocabulary of the text is large, the vector dimension of one-hot encoding is very large, resulting in a dimensional disaster. The one-hot encoding ignores the connection between different words, and there is a “vocabulary gap.” To address these shortcomings of one-hot coding, some researchers have proposed distributed vector representations. Among them, the word embedding method based on skip-gram and CBOW model are the most representative. Skip-gram uses the training data in the corpus to predict the possible words near the headword, while CBOW uses several nearby words to predict the possible headwords of these words. In this study, in order to compare the impact of different word embedding methods on the accuracy of the model, we adopt two word embedding methods, respectively.

#### 3.2.3. Contextual Semantic Modeling

RNN has no ability to filter information; it stores all the context information. While LSTM is a variant of RNN, a higher-level RNN can selectively store information. Ordinary RNN has only the middle memory unit, while LSTM has three carefully designed gate structures to control information memory and forgetting at every moment. Its main structure is shown in Figure 4.

Forgetting gate reads *h*_*t*−1_ and Xt, output a value between 0 and 1 by activating the sigmoid function.

(1) $$\begin{array}{c} f_{t}=\sigma \left(w_{f}\left[h_{t-1},X_{t}\right]+b_{f}\right), \end{array}$$

where *w*_*f*_ represents the weight, *b*_*f*_ represents the offset, and *σ* represents the activation function.

Input gate determines what value will be updated.

(2) $$\begin{array}{c} i_{t}=\sigma \left(w_{i}\left[h_{t-1},X_{t}\right]+b_{i}\right), \end{array}$$

(3) $$\begin{array}{c} a_{t}=\tanh\left(w_{a}\left[h_{t-1},X_{t}\right]+b_{a}\right), \end{array}$$

(4) $$\begin{array}{c} C_{t}=C_{t-1}*f_{t}+i_{t}*a_{t}, \end{array}$$

where *w*_*i*_ and *w*_*a*_ represent the weight, *b*_*i*_ and *b*_*a*_ represent the offset, and *σ* represents the activation function.

Output gate is utilized to determine the output content.

(5) $$\begin{array}{c} o_{t}=\sigma \left(w_{o}\left[h_{t-1},X_{t}\right]+b_{o}\right), \end{array}$$

(6) $$\begin{array}{c} h_{t}=o_{t}*\tanh\left(C_{t}\right), \end{array}$$

where *w*_*o*_ represents the weight, *b*_*o*_ represents the offset, and *σ* represents the activation function.

Bidirectional LSTM (BI-LSTM) is a network that combines forward LSTM and backward LSTM at the same time and splices the output of each LSTM unit into the final output, so that the output of each unit contains the complete context information of each word in the input comment, and its model structure is shown in Figure 5.

When the context vector *X* = {*x*_1_, *x*_2_, ⋯, *x*_*n*_} of the comment is input, the hidden layer state output of the forward LSTM ${\overset{⟶}{h}}_{t}$ can be expressed as

(7) $$\begin{array}{c} {\overset{⟶}{h}}_{t}=\text{LSTM}\left(x_{t},{\overset{⟶}{h}}_{t-1}\right). \end{array}$$

Similarly, the hidden layer state output of the backward LSTM can be expressed as

(8) $$\begin{array}{c} {\overset{⟵}{h}}_{t}=\text{LSTM}\left(x_{t},{\overset{⟵}{h}}_{t-1}\right). \end{array}$$

The hidden layer state output of BI-LSTM at time t *h*_*t*_ can be expressed as follows:

(9) $$\begin{array}{c} h_{t}=\left[{\overset{⟶}{h}}_{t},{\overset{⟵}{h}}_{t}\right]. \end{array}$$

The hidden layer state *h*_*t*_ is the memory fragment input in the next stage, which is recorded as *m*_*j*_, so the total input *M* in the next stage can be expressed as follows:

(10) $$\begin{array}{c} M=\left\{m_{1},m_{2},\cdots ,m_{j},\cdots ,m_{n}\right\}. \end{array}$$

#### 3.2.4. Sentiment Representation

The session is utilized to adaptively extract useful information from memory, and each computational layers contains an attention layer and LSTM units, whose structure is illustrated in Figure 6. The attention mechanism makes the model focus on the key information among many input information, reduce the attention to other information, or even ignore other information, and improve the efficiency and accuracy of task processing.

The priori knowledge *y*_*i*_ is first input, and the sentiment vector is extracted from the memory *M* adaptively after weighting the memory slice through the attention layer; then, the output of the attention layer and the priori knowledge is input to the LSTM unit to achieve selective enhancement or forgetting of the priori knowledge, and its output is used as the input of the next computational layer; the priori knowledge is continuously updated through multiple computational layers, and the output vector in the last layer is the sentiment representation of the teaching comments about the a priori knowledge.

In the attention layer, for each memory fragment *m*_*j*_, a feedforward neural network is utilized to compute its semantic relevance to prior knowledge, calculated as follows:

(11) $$\begin{array}{c} h_{j}^{t}=\tanh\left(W_{\text{att}}\left[m_{j},y_{i}^{t-1}\right]+b_{\text{att}}\right), \end{array}$$

where *W*_att_ is the weight matrix, [*m*_*j*_, *y*_*i*_^*t*−1^] is the splicing vector of memory slices *m*_*j*_ and *y*_*i*_^*t*−1^, and *b*_att_ is the offset.

The weight of attention layer can be calculated as follows:

(12) $$\begin{array}{c} \alpha_{j}^{t}=\frac{\exp\left(h_{j}^{t}\right)}{\sum_{j=1}^{n}\exp\left(h_{j}^{t}\right)}. \end{array}$$

Obviously, 0 ≤ *α*_*j*_ ≤ 1 and ∑_*j*=1_^*n*^*α*_*j*_ = 1.

#### 3.2.5. Sentiment Recognition

The output vector *y*_*i*_^*K*^ of the last computing layer is the final emotional feature *y*_*o*_, which is input into a softmax classifier for emotional classification:

(13) $$\begin{array}{c} p_{g}=\frac{\exp\left(W_{s}\cdot y_{o}+b_{s}\right)}{\sum_{g=1}^{G}\exp\left(W_{g}\cdot y_{o}+b_{s}\right)}, \end{array}$$

where *G* is the number of emotional categories and *p*_*g*_ is the probability of being classified as category *g*.

The model is trained using an end-to-end backpropagation algorithm, and the cross entropy is used as the loss function. L2 regularization is added to avoid overfitting of the model during the training process. Train the model in a supervised manner by minimizing the loss function and the regularization term, and its loss function is as follows:

(14) $$\begin{array}{c} \text{Loss}=-\underset{\left(s,a\in D\right)}{\sum }\underset{g\in G}{\sum }y_{k}^{g}\left(s,a\right)\cdot \log\left(p_{k}^{g}\left(s,a\right)\right)+\lambda {\left\|\theta \right\|}^{2} \end{array}$$

where *D* is the training dataset, *y*_*k*_^*g*^(*s*, *a*) is the actual emotion category of the comment in a certain aspect, *p*_*k*_^*g*^(*s*, *a*) is the predicted emotion category of the comment in a certain aspect, *λ* is L2 regularization weight, and *θ* is a set of all trainable parameters in the model.

### 3.3. Teaching Evaluation Based on LSTM and Comprehensive Indicators

This study combines the teaching scoring in Section 3.1 with the emotional classification results of teaching comment in Section 3.2 as the input data of TE model and realizes the teaching evaluation of the course through the LSTM model. In this study, one-hot encoding and Word2vec encoding are adopted for course comments to compare the impact of different word embedding methods on model performance, and one-hot encoding is utilized for course grades. All data need to be normalized before input. The whole TE model is shown in Figure 7.

## 4. Empirical Analysis

### 4.1. Data Collection and Analysis

The data used in this research are the teaching evaluation data of students in the course of mental health education from 2011 to 2021 provided by Zhengzhou College of Finance and Economics. And the data have been encrypted with the teacher's work number, course number, course name, student number, and student name, so that the privacy of students and teachers will not be violated. In addition to the comprehensive scores given by students to teachers, the data also includes students' text evaluation of teachers. The expected score has been given by the educational administration supervision experts. A total of 52106 valid text evaluation data and corresponding scores were obtained in this paper. The dataset are separated into training set corpus and test set corpus according to the ratio of 8 : 2. After a simple preprocessing, the aspect labels and sentiment labels of the comments need to be manually labeled. The statistical information of the labeled TE dataset is shown in Figures 8–10.

In Figure 8, the abscissa indicates the five first-level indicators of teaching attitude, teaching effectiveness, teaching method, lecture effect, and psychological improvement, respectively. The red bar indicates the proportion of data with positive emotion, the blue bar indicates the proportion of data with neutral emotion, and the green bar indicates the proportion of data with negative emotion. The abscissa of Figure 9 is the same as that of Figure 10. In Figure 10, the abscissa indicates the three second-level indicators of positive psychological changes, extracurricular extension, and Marxist perspective on the problem in psychological improvement, respectively. The solid blue line represents students majoring in Marxist, the solid red line represents students from other majors, and the dotted line indicates the mean. It is apparent that Marxism majors scored higher in psychological improvement than other majors because Marxism majors received higher scores in the area of “Marxist perspective.”

### 4.2. The Accuracy of ASBA on Teaching Comment Text

#### 4.2.1. The Impact of the Word Embedding Dimension on the Model Accuracy

The paper investigates the effect of different dimensions of word vectors and different numbers of computational layers on the sentiment classification results and compares the effect of PI-DMN model sentiment analysis with different word vector dimensions and number of computational layers, the accuracy of which is shown in Figure 11. The model adopts one-hot word encoding and uses a dataset labeled with first-level aspect labels.

It can be seen that with the increase of word vector dimension, the accuracy of classification gradually improves, but the amount of increase gradually decreases. This is because the high-dimensional word vector contains richer information, which can model words more accurately. However, when the word vector dimension is high enough, the increase of effective semantic information decreases, resulting in a slow increase in accuracy. With the increase of the number of computing layers, the effect of emotional classification of the model has also been significantly improved, reaching the maximum at the fourth layer. When the computing layer reaches the fifth and sixth layers, the performance has not increased significantly. This is because the increase of computing layer can repeatedly extract the emotional information in memory, making the emotional classification more accurate. At the same time, it will also cause the loss of semantic information in the transmission process and finally make the performance reach a balance.

#### 4.2.2. The Impact of Prior Knowledge and Word Embedding Method on Classification Accuracy

This study compares the accuracy of emotion classification under different prior knowledge, that is, “aspect + emotion,” “emotion,” and no prior knowledge, which are recorded as ABSAPI-DMN, EPI-DMN, and NPI-DMN, respectively. And we compares the model classification effects of different word embedding methods, that is, one-hot encoding and Word2vec encoding. Word2vec embedding uses 100 dimensional word vectors, one-hot embedding uses 3-bit coding, and the calculation layer is 4 layers. The results of model performance are shown in Figure 12.

It can be seen that the model with prior knowledge has a certain improvement in accuracy and macro F1 than the model without prior knowledge, and the model with only emotional tags has a higher accuracy than the model with both aspect tags and emotional tags. This is because the model is equivalent to a model that needs to answer a more complex question, so the effect is not as good as a model that only judges emotional tendencies. At the same time, it can be seen that the Word2vec embedding method is obviously not as effective as the one-hot embedding method, because when the prior knowledge is embedded with Word2vec, there are more model parameters and less training datasets, resulting in serious under fitting. Therefore, this paper selects one-hot encoding to realize word embedding.

#### 4.2.3. Comparison of Different Models in TE

We compared the classification accuracy of PI-DMN model with other commonly used classical models in five aspects of student evaluation, and the results are shown in Figure 13. The model adopts the one-hot word encoding method and uses the dataset labeled with the first-level aspect label, and the number of computational layers is set to 4 layers.

It is apparent that the PI-DMN model proposed in this paper has a better classification effect than the existing methods, especially it can obtain aspect-level sentiment analysis for different teaching aspects, which fully reflects the superiority of the PI-DMN to the emotional analysis of students' teaching evaluation. CNN is not good at dealing with long sentences, and it is prone to ignore the context dependent information of comments, resulting in general performance. While AT-LSTM can effectively excavate the context-sensitive information in comments and utilize the attention mechanism to give weights to specific words, so the emotional classification results are better.

### 4.3. Verification of TE Based on DL

A total of 729 evaluations of mental health courses were obtained for this study, including 48 for Marxist students, which is a small sample size. Therefore, this paper trained the model with data from all students and used a fivefold cross validation approach.

#### 4.3.1. The Impact of Training Data on the Accuracy of Model

This paper investigates the accuracy of model prediction under different training dataset, which is course scoring data only, teaching evaluation text data only, and the dataset used in this paper. The prediction results are shown in Figure 14. The model adopts the one-hot word coding method, and the dataset with teaching evaluation text is labeled with the first-level aspect label, and the number of computational layers is 4.

The ordinate indicates the average value of prediction error. Clearly, the dataset used in this paper has a much smaller prediction error, and the model using only the course scoring data has the lowest accuracy. This is because students are perfunctory in scoring the course, which leads to inaccurate data and cannot objectively reflect the true evaluation of the course.

#### 4.3.2. The Impact of Label Granularity on the Accuracy of Model

We compared the accuracy at different fine granularity of aspect labels, which are no aspect label, first-class index labeling for aspect labels of datasets, and second-class index labeling for aspect labels of datasets. The prediction results are shown in Figure 15.

The red bar indicates the first-level metric labeling of the dataset aspect labels, the green bar indicates the second-level metric labeling of the dataset aspect labels, and the blue bar indicates no aspect labels. It is apparent that the accuracy of the model is higher when aspect labels are present, but the accuracy of the model decreases instead when the dataset has more fine-grained second-level aspect labels labeled. This is because the more aspect labels, the more complex problems the model has to deal with, resulting in a reduction in accuracy with the same amount of data.

## 5. Conclusions

A fair and objective evaluation of teachers' curriculum is an important method to stimulate teachers' enthusiasm for work, guide teachers to improve teaching methods, and promote teaching quality. Curriculum is the basic unit of teaching, so improving the quality of curriculum is a very important measure to ensure the quality of education. Schools should regularly organize and carry out teaching evaluation to objectively and fairly evaluate the quality and effect of teachers' classroom teaching as far as possible, so as to promote the growth of teachers. Data mining and text mining have been extensively adopted in the field of education, but the application on student feedback needs further research. The existing information processing method for students' evaluation of teaching adopts the method of averaging all scores of the same teacher, and no processing measures are taken for students' written feedback.

Based on DL, this study establishes a SET model of mental health curriculum considering the influence of Marxism, considering students' teaching evaluation scores and curriculum evaluation texts comprehensively. Firstly, five first-level indicators and corresponding second-level indicators considering the promotion of Marxism to mental health for evaluating mental health courses are proposed. Based on the DMN model, the PI-DMN model is proposed, which realizes the emotional analysis of teaching evaluation in the five first-level indicators. Through four processes (text preprocessing and word embedding, contextual semantic modeling, sentiment representation, and sentiment recognition), the emotional analysis of students' curriculum evaluation text is realized. Finally, the LSTM model is trained by the dataset combined students' scoring and sentiment analysis results to realize TE. The data analysis shows that students majoring in Marxism have higher scores in the secondary index psychological improvement. And the results of the empirical analysis show that the accuracy of teaching evaluation can be improved by considering the sentiment analysis of evaluation texts, and the accuracy of teaching evaluation can also be improved to a certain extent after aspect labeling of the dataset, but the prediction accuracy of the model decreases with the increase of labeling fineness.

## Figures and Tables

**Figure 1:** The structure of MN.

**Figure 2:** The structure of the four-layer DMN.

**Figure 3:** The structure of the PI-DMN model.

**Figure 4:** The structure of LSTM.

**Figure 5:** The structure of BI-LSTM.

**Figure 6:** Sentiment representation modular.

**Figure 7:** Flowchart of TE modeling.

**Figure 8:** Statistical information on sentiment labels and aspect labels.

**Figure 9:** Scoring on different aspect labels.

**Figure 10:** Scores of students majoring in Marxism and other majors in psychological improvement.

**Figure 11:** The impact of the word embedding dimension on the model accuracy.

**Figure 12:** The impact of prior knowledge and word embedding method on model performance.

**Figure 13:** The performance of different models in emotion classification.

**Figure 14:** The impact of training data on model performance.

**Figure 15:** The impact of label granularity on model performance.

**Table 1:** Teaching evaluation indicators of mental health course.

First-level indicators	Second-level indicators	Second-level indicator explanation
Teaching attitude	Enthusiasm	Teacher is passionate about teaching
	Lesson preparation	The teacher carefully prepares the course
	Punctuality	The teacher is very punctual
Teaching effectiveness	Passion and vitality	The teacher's lectures are full of enthusiasm and vitality
	Interest	Teacher's lectures are interesting
	Readability	The teacher explained the course very clearly
Teaching method	Teacher-student interaction	Teacher encourages students to express personal opinions
	Encourage dissent	Teacher encourages students to question themselves
	Fair assessment	The teacher's course assessment method is very fair
	Enlightenment	The teacher's lessons help me to think positively
Lecture effect	Course interest	Students are very interested in the course
	Course benefits	Students learned a lot during the course
	Problem-solving	Improve students' problem-solving skills
Psychological improvement	Positive psychological changes	Students have positive changes in their psychology
	Extracurricular extension	Students have practical actions to adjust their psychological state
	Marxist perspective on the problem	Students can use Marxist philosophy to solve troublesome emotions

## Data Availability

The labeled dataset used to support the findings of this study is available from the corresponding author upon request.
